# Investigation of Influencing Factors on the Prevalence of Retinopathy in Diabetic Patients Based on Medical Big Data

**DOI:** 10.1155/2022/2890535

**Published:** 2022-04-12

**Authors:** Lei Yang, Qin Qi, Fangjiang Zheng, Yanqiang Wei, Qiaoe Wu

**Affiliations:** ^1^Ophthalmology, Nanjing Tongren Hospital Southeast University, Nanjing, 211102 Jiangsu, China; ^2^Department of Endocrinology, The Third People's Hospital of Gansu Province, Lanzhou 730000, China; ^3^Publicity Department, Gansu Provincial Hospital of Traditional Chinese Medicine, Lanzhou, 730050 Gansu, China; ^4^Key Laboratory of Remote Sensing of Gansu Province, Northwest Institute of Eco-Environment and Resources, Chinese Academy of Sciences, Lanzhou 730000, China; ^5^Ophthalmology, Zhuanglang County People's Hospital, Pingliang, 744600 Gansu, China

## Abstract

As one of the most important organs of human beings, the eyes can receive external visual information and play an important role in perception. Therefore, the method of maintaining eye health is a problem that people pay attention to. Omental disease is one of the most serious microvascular complications in diabetic patients, and it is also the main cause of blindness in patients. The purpose of this article is to investigate the main factors that influence the prevalence of retinopathy in diabetic patients based on medical big data. In this article, a method for investigating the causes of the incidence of retinopathy in diabetic patients based on medical big data is proposed, and a questionnaire survey method and other methods are used for experimental investigation. Combining the data in the figure in the experiment in this article, it can be seen that among diabetic patients, the prevalence of diabetes in men is 12.4%, and the prevalence of diabetes in women is 8.4%. From the data in the figure, it can be known that the rate of retinopathy caused by various factors is between 5% and 7%, and the total prevalence of retinopathy is 47.5%. There are many factors affecting the prevalence of retinopathy in diabetic patients, such as the duration of diabetes, urinary albumin index, glycosylated hemoglobin index, and fasting blood glucose level; various factors lead to an increase in the prevalence of retinopathy in diabetic patients. The results show that there are many factors affecting the prevalence of retinopathy in diabetic patients, so patients should pay attention to exercise, control their diet, and prevent retinopathy.

## 1. Introduction

Patients with diabetic retinopathy are getting younger and younger. There are more than 100 million diabetic patients. Among adult diabetic patients, the prevalence of diabetic retinopathy is 24.7%~37.5%, and the number of patients has reached more than 30 million. Therefore, the screening and prevention of diabetes is particularly important. The doctor's diagnosis mainly relies on clinical experience, while the traditional research method is to analyze the main physiological characteristics of retinopathy in a large amount. With the deepening of science and technology in the medical industry, society has carried out a series of reforms in medical-related fields. Medical big data comes from clinical diagnosis, health checkups, health websites, medical research, and other aspects. These data contain rich information. In today's era of rapid development of big data, almost all walks of life can use massive data to further improve the development of the industry, as an important part of the big data system, medical big data is a valuable resource in the medical and health field. It is discussed based on the medical and health field, including life related to maintaining the health of the body. Medical big data is no exception in the medical and health field related to people's health. When traditional medical cases are stored in the form of big data, medical institutions can extract medical data of related cases or related patients in a timely manner during consultation and treatment. In this way, doctors can be given more data guidance, so that patients can enjoy more accurate diagnosis and treatment and considerate services. Medical cause has a great impact on people's physical quality. The better the medical cause, the better people's physical quality will be. Kumar et al. found that the main cause of more and more people suffering from blindness is diabetic retinopathy. It has been found that corticosteroid therapy plays a major role in the treatment of diabetic retinopathy. Therefore, the most important thing is to develop new drugs. In addition, it is found that antiangiogenic agents play a great role in diabetic retinopathy [1]. Ting et al. found that diabetic retinopathy is the leading cause of loss of vision. Timely detection and timely treatment can prevent early diabetic retinopathy. Timely reporting to the hospital and reporting to doctors can prevent diabetes-related complications. With the increasing prevalence of diabetes and DR, the cost of medical industry will also increase. Therefore, timely prevention and treatment can solve this problem [2]. Leasher et al. estimate the global regional trends from 1990 to 2010, especially the number and prevalence of visually impaired diabetic retinopathy (DR), as a complication of the rapid global trend of diabetes, which is essential for health planning purposes. The number of people with visual impairment due to DR is increasing worldwide, and it accounts for an increasing proportion of all causes of blindness, and the age-standardized prevalence of DR-related blindness is increasing. One out of 39 blind persons is blind due to DR, and one out of 52 visually impaired persons has visual impairment due to DR [3]. Taylor-Phillips et al. found that if the screening interval of UK diabetic retinopathy is less than 1 year, the safety of people can be improved. They searched 10 databases. They made a comparative experiment with economic modeling research. They found that the age of these patients was at different stages, so diabetes patients had little relationship with age. They also reported the incidence and progress of DR. They obtained data on 262541 patients, of which at least 228649 (87%) had type 2 diabetes. There are no randomized controlled trials. The study concluded that there is almost no difference in the clinical results of low-risk patients who are screened for 1 year or 2 years each year [4]. Wang et al. found that little is known about his risk of developing diabetic retinopathy. He tried to determine the risk factors for DR in adolescents with diabetes, compare the DR rates of adolescents with T1DM and adolescents with T2DM, and assess whether to comply with the DR screening guidelines advocated by the Ophthalmological Society. The Pediatric Society and the Diabetes Association fully documented the adolescents with DR. A retrospective observation longitudinal cohort study was designed, and a multivariate Cox proportional hazard regression model was determined [5]. Morrison et al. found that the prevalence of gestational diabetes is also increasing. Of the 120 pregnancies, 1 had diabetic retinopathy, and diabetic retinopathy led to blindness among pregnant women and a greater risk of diabetic retinopathy during pregnancy. There are many reasons for gestational diabetic retinopathy, such as diabetes duration, blood sugar control level, and hypertension. They studied a range of treatments and further studied on how to reduce the prevalence [6]. Sebaa et al. found that the proliferation of medical devices and clinical applications that produce a large amount of data has brought great problems to manage, process, and mine a large amount of data. In fact, the traditional data warehouse framework cannot effectively manage the number, type, and speed of current medical applications. Therefore, some data warehouses face many problems and challenges in medical data. New solutions have emerged, and Hadoop is one of the best examples, which can be used to process these medical data streams. However, without efficient system design and architecture, these attributes have no significance and value for medical managers. In this paper, the architecture based on Hadoop and the conceptual data model for designing medical big data warehouse are given [7]. Price and Cohen found that big data has become a universal slogan for medical innovation. The rapid development of machine learning technology and artificial intelligence, from resource allocation to diagnosis of complex diseases, is expected to revolutionize medical behavior. However, big data brings great risks, including major issues related to patient privacy. Here, the legal and ethical issues that big data brings to the private lives of patients are summarized. Among other topics, they also discussed how to better consider health privacy, fairness, consent, the importance of patient governance, differences in data use, and methods to deal with data infringements. Finally, an overview of possible regulatory systems in the future is explained [8]. Through the experimental analysis of scholars, it can be seen that there are more and more people suffering from diabetic retinopathy, regardless of whether it is a low-age group or a high-age group, but the factors are not yet clear. How to prevent diabetic retinopathy is also a major problem today.

The innovation of this article is as follows: (1) investigate and research the factors affecting the prevalence of retinopathy in diabetic patients based on medical big data through investigation and research methods, study the factors that affect the prevalence of retinopathy in diabetic patients by medical big data, and then discuss how to prevent retinopathy in diabetic patients in the first place and (2) using deep-supervised residual network algorithm to popularize relevant medical knowledge and reduce the prevalence.

## 2. Deeply Supervised Residual Network Algorithm

### 2.1. In-Depth Supervision Network Method

Deep residual network is an improved convolutional neural network, which reduces the difficulty of model training by introducing an identity path. Under the effect of the identity path, the difficulty of training network parameters is greatly reduced, so that it is easy to train a good deep learning model. This article will give a detailed introduction to the proposed diabetic retinopathy severity, classification depth, and supervised residual network [9]. Traditional CNN networks usually face the following problems: the transparency of the influence of the features learned by the middle layer of the network on the overall classification effect of the network and the discriminativeness of the features learned by each layer of the network (especially the shallow layer) [10]. In response to these problems, this paper proposes a deep supervision network, and the structure of the network is shown in Figure 1:

As shown in Figure 1, the implementation provides direct supervision on the feature learning of the hidden layer, instead of relying on the error backpropagated from the final classification layer to guide the learning of the hidden layer like the traditional CNN network [11]. The introduction of these additional deep supervision objective functions mainly brings the following two benefits: for shallower networks, additional regularization items can be provided during network training, thereby improving the discriminativeness of learned features; for deeper networks, to some extent, the problem of “gradient disappearance” in network training can be solved [12] and the performance of the network can be improved.

In view of the traditional CNN network, as the number of network layers increases, “gradient disappearance” may occur during network training, and the performance of the network is obviously degraded. This paper proposes a new network structure of “deep residual network” composed of “residual units” stacked, in which the structural diagram of the residual unit is shown in Figure 2:

As shown in Figure 2, unlike the traditional network directly learning the expected mapping, ResNet learns the residual mapping through residual learning and the introduction of skip connections in the network. It makes the optimization and training of extremely deep networks easier, so that the performance of the network is greatly improved [13].

It also uses a convolutional neural network. Convolutional neural network is a neural network designed specifically for image recognition problems, which imitates the multilayer process of human image recognition to further abstract judgment. The specific structural parameters of the network are shown in Table 1:

As shown in Table 1, this paper can define a “multicategory balanced cross-entropy loss function” [14], in which the concepts of “side output layer” and “fusion layer” are expressed by

(1) $$\begin{array}{c} \varsigma_{\text{side}}^{i}\left(A,a^{I}\right)=\frac{1}{N}\beta^{c}\log a^{i}, \end{array}$$

(2) $$\begin{array}{c} \varsigma_{\text{fuse}}^{i}\left(A,a^{\text{fuse}},a\right)=-\frac{1}{N}\beta^{c}\log\left(\rho_{n}^{c}\left|X_{n}\right.\right). \end{array}$$

Taking into account the prediction loss of the “side output layer” and the “fusion layer,” the overall loss function of the network is shown:

(3) $$\begin{array}{c} \varsigma_{\text{fuse}}^{i}\left(A,a^{\text{fuse}},a\right)=\overset{s}{\underset{i=1}{\sum }}\alpha_{i}\varsigma_{\text{side}}^{i}\left(A,a^{i}\right). \end{array}$$

In the formula, *S* represents the number of “side output layers”; *a*^*i*^ represents the weight of the *i*-th “side output layer” prediction loss; *ς*_fuse_^*i*^ represents the weight of the “fusion layer” prediction loss. In the end, the training of the network is

(4) $$\begin{array}{c} \left(A,a^{\text{fuse}},a\right)=\arg\min\left(A,a^{\text{fuse}},a\right). \end{array}$$

When training the network, conventional stochastic gradient descent is used to optimize the objective function shown in formula (4).

### 2.2. Decision Tree Method

Decision tree is a process of classifying data through a series of rules. It provides a rule-like method of what value will be obtained under what conditions. Decision trees are divided into classification trees and regression trees. Classification trees are used as decision trees for discrete variables, and regression trees are used as decision trees for continuous variables. The growth of decision trees mainly depends on information entropy and information collection algorithms [15]. The conditional probabilities of all channels constitute matrix *P*(*U*|*V*), which is called the information transmission probability matrix, which is expressed as

(5) $$\begin{array}{c} P\left(U\left|V\right.\right)=P\left(u_{1}\left|v_{1}\right.\right)LP\left(u_{I}\left|v_{1}\right.\right). \end{array}$$

The information transmission probability matrix has properties such as

(6) $$\begin{array}{c} \underset{i}{\sum }P\left(u_{i}\left|v_{j}\right.\right)=1. \end{array}$$

The amount of information in the information *u*_*i*_ sent by the source is

(7) $$\begin{array}{c} I\left(u_{i}\right)=\log_{2}\frac{1}{p\left(u_{i}\right)}=-\sum p\left(u_{i}\right)\log_{2}p\left(u_{i}\right). \end{array}$$

Information entropy represents the mathematical expectation of all information, and the information entropy of source *U* is defined as

(8) $$\begin{array}{c} \text{Ent}\left(u\left|v\right.\right)=\sum p\left(u_{i}\right)\log_{2}p\left(u_{i}\right). \end{array}$$

In order to solve this problem, the decision tree method uses the information acquisition rate as a selection criterion. The expression is ∑_*i*_*P*(*u*_*i*_|*v*_*j*_) = 1. If the information entropy is too large, the information acquisition rate will decrease, and multiple influences will be excluded from the classification. The decision tree method is to select the variable with the largest information acquisition rate as the best combination variable [16].

### 2.3. Postpruning Algorithm

There are two methods of decision tree pruning: prepruning and postpruning. The difference between the two is that prepruning participates in the construction of the decision tree, and postpruning is pruning from the bottom up after the decision tree is constructed. The important problem of the postpruning algorithm is the design error and the method of setting the pruning standard. In the error design, the decision-making method is to use the training samples to directly guess the error, and the default reliability is 75%; the basic idea is as follows [17]:

Suppose the *i*-th node contains *M*_*i*_ predicted values, including *n*_*i*_ wrong predictions, and then, the error is *H*_*I*_ = *n*_*i*_/*M*_*i*_. Assuming an approximate normal distribution, the interval estimation of the true error of the *I*-th node is set, and the confidence level is set to 1, and then, it is

(9) $$\begin{array}{c} P=\left[\frac{h_{i}-e_{i}}{\sqrt{h_{i}\left(1-h\right)/M_{I}}}≺1\right]=1-\alpha . \end{array}$$

In the formula, *h*_*i*_ − *e*_*i*_ is the critical value. Therefore, according to formula (9), the upper limit of confidence for the true error of the *I*-th node is pessimistically estimated as

(10) $$\begin{array}{c} \overset{k}{\underset{i=1}{\sum }}p_{i}e_{i}≻e. \end{array}$$

In the setting of pruning criteria, C5.0 is based on the “error reduction” method that determines whether to prune based on error estimates.

A certain node *j* in the hidden layer of the three-layer artificial neural network graph consists of an adder and an activation function, as shown in Figure 3:

As shown in Figure 3, ANN contains multiple hidden layers, and the nodes of the hidden layer and the output layer are processed by the adder and the activation function.

Functional formula usually has the following four methods, which are introduced below.

The [0,1] type step function is

(11) $$\begin{array}{c} f\left(U_{j}\right)=\left\{\begin{array}{c} 1,u_{j}≻0\\ 0,u_{j}\leq 0 \end{array}\right\}. \end{array}$$

The [-1,+1] type step function is

(12) $$\begin{array}{c} f\left(U_{j}\right)=\left\{\begin{array}{c} 1,u_{j}≻0\\ -1,u_{j}\leq 0 \end{array}\right\}. \end{array}$$

The (0,1) type Sigmoid function is

(13) $$\begin{array}{c} f\left(U_{j}\right)=\frac{1}{1+e^{-u_{i}}}. \end{array}$$

The (-1,1) type Sigmoid function is

(14) $$\begin{array}{c} f\left(U_{j}\right)=\frac{1-e^{-u_{i}}}{1+e^{-u_{i}}}. \end{array}$$

The graph of the activation function is shown in Figure 4:

As shown in Figure 4, the mapping of the calculation result of the adder to the range of a specific value is a function of the activation function. The general procedure for ANN establishment is (1) prepare data, (2) determine the ANN structure, and (3) determine the weight of the ANN. The complexity of the network structure determines the difficulty of ANN processing [18]. Based on the above expressions, any observation value should satisfy

(15) $$\begin{array}{c} b_{i}\left(b+W^{T}a_{i}\right)\geq d. \end{array}$$

The basis for support vector classification to have the best generalization error is to ensure that the goal of hyperplane solution is to maximize *d*, as shown in Figure 5:

As shown in Figure 5, the objective function of the optimization problem is a quadratic function, and the constraints are linear. This is a convex optimization problem, which can be solved by the standard Lagrangian multiplier method [19].

### 2.4. Confusion Matrix Method

Confusion matrix is a useful tool for analyzing classifiers to identify tuples of different classes. For a binary classification problem of yes and no, the prediction may produce 4 different results, as shown in Table 2:

As shown in Table 2, in practice, 30% is generally reserved for testing, and the remaining 70% is used for training, but these samples may not be representative. Therefore, in random sampling, each class in each data set must have a corresponding proportion [20].

The mean square error is expressed by MSE. The smaller the MSE value, the smaller the mean square error, and the higher the accuracy of the prediction model:

(16) $$\begin{array}{c} \text{MSE}=\frac{{\left(p_{1}-b_{1}\right)}^{2}+\cdots +{\left(p_{n}-b_{n}\right)}^{2}}{n}. \end{array}$$

RMSE is very sensitive to the error response of extreme points and can well reflect the accuracy of the prediction model:

(17) $$\begin{array}{c} \text{MSE}=\sqrt{\frac{{\left(p_{1}-b_{1}\right)}^{2}+\cdots +{\left(p_{n}-b_{n}\right)}^{2}}{n}}. \end{array}$$

In addition, the mean square error tends to exaggerate the influence of outliers, while the absolute error has no such effect:

(18) $$\begin{array}{c} \text{MAE}=\frac{\left|p_{1}-b_{1}\right|+\cdots +\left|p_{n}-b_{n}\right|}{n}. \end{array}$$

The relative square root error is the square root of the relative square error, denoted as RRSE:

(19) $$\begin{array}{c} \text{RRSE}=\frac{{\left(P_{1}-b_{1}\right)}^{2}+\cdots +{\left(P_{N}-b_{N}\right)}^{2}}{{\left(b_{1}-b_{1}\right)}^{2}+\cdots +{\left(b_{n}-b\right)}^{2}}. \end{array}$$

The relative absolute error is actually the standardization of the absolute error, which is recorded as RAE. These three relative error measures are all normalized using the simple predictor error of the predicted average, which is

(20) $$\begin{array}{c} \text{RAE}=\frac{\left|P_{1}-b_{1}\right|+\cdots +\left|P_{n}-b_{n}\right|}{\left|b_{1}-b\right|+\cdots +\left|b_{n}-b\right|}. \end{array}$$

### 2.5. Trajectory Algorithm

Orbital data has become more and more important in the research and application of daily big data. With the advancement of wireless communication and sensor technology, the acquisition of orbits has become easier. Among them, the movement trajectory data is a type of position-related trajectory data, and a continuous trajectory is generated when a moving object moves. Through wireless signal propagation and sensor information sampling, multiple discrete track points can be obtained. The track point information usually contains the position, and these track points are located in the time series together with time or other attributes to approximate the current track of the moving object. Therefore, the moving track data is also a kind of time series data, and the definition of the track can be

(21) $$\begin{array}{c} \text{Traj}=\left\{\left(u_{2},t_{1}\right),\left(u_{2},t_{1}\right),\cdots \left(u_{i},t_{i}\right)\right\}. \end{array}$$

A typical trajectory is shown in Figure 6:

As shown in Figure 6, the general movement trajectory data includes vehicle GPS movement trajectory, animal movement trajectory, and cluster movement trajectory. Various trajectories have been utilized in their respective research and application fields, and they have made certain contributions in various fields. This article is based on the trajectory generated by the mobile device when receiving information. Using this data, you can discuss and investigate the similarity of the trajectory.

## 3. Experiment

### 3.1. Experiment of Decision Tree Algorithm Based on Medical Big Data

The incidence of diabetes is about 11%. Diabetes is a common clinical metabolic disease, which is mainly manifested as chronic hyperglycemia, which is caused by defects in insulin secretion or utilization. Diabetes is getting younger and younger, and its prevalence is increasing year by year. It has become one of the leading causes of blindness. Therefore, popularization and promotion of screening, early detection, early diagnosis and treatment, and long-term follow-up can prevent patients from blindness. With the aid of modern computer technology in the early stage of DR screening, the automatic examination and classification of the disease is realized as a large-scale screening method to promote the improvement of the potential limit between the results of the automated detection system under the ideal model and the real clinical effect, maximize the detection effect of DR, detect the early stage in time, and slow down or even avoid the development of visual impairment.

At present, the prevalence and incidence of diabetes are on the rise in the world. In recent years, due to the westernization of lifestyle, the aging of the population, the rising obesity rate, and other reasons in China, the prevalence of diabetes has also been increasing rapidly. In addition, some diabetic patients failed to be diagnosed because they did not pay attention to physical examination. Diabetes can cause metabolic disorders of carbohydrates, fats, and proteins, leading to multisystem functional damage, various acute and chronic complications, and life-threatening in severe cases. Using 10 times of 10-fold cross-validation, under different integration algorithms, the integration scale is set to 20, 30, 40, 50, and 60, two methods of pruning and unpruning are used to compare the decision tree integration, and the average prediction accuracy is used as the comparison data. The experimental comparison results under different pruning strategies are shown in Tables 3 and 4:

Through the comparison of Tables 3 and 4, it is found that under the pruning strategy, only Bagging is 87.754, Rotation Forest+C4.5 reaches 94.132, and C4.5 is the highest with 97.321. The Rotation Forest integration algorithm has fewer failures, and the AdaBoostM1 and MultiBoostAB integration algorithms all fail. It shows that under this data set, the classification accuracy of the base classifier has reached better, and the improvement effect of the integrated algorithm is not very obvious. With the increase of the integration scale, some integration algorithms have a downward trend, and the Rotation Forest integration algorithm does not show any improvement advantages in this case. Only when the integration scale is 40, it is higher than the classification accuracy of the base classifier.

This paper compares and analyzes the sensitivity index and specificity of the integrated classifier under the decision tree algorithm, as shown in Figure 7:

As shown in Figure 7, under the complex clinical data set, the sensitivity index of the ensemble classifier is between 20 and 30, and there is not much fluctuation, and the highest is only 67 once. However, the specificity is much higher than the base classifier, with the lowest being 35 and the highest being 70. It shows that the integrated algorithm improves the ability to predict nonpatients and also improves the total ability of predicting nonpatients and patients to a certain extent.

Basically, patients with diabetes will have metabolic disorders of body fat, carbohydrates, and protein, which may be acute or chronic long-term accumulation. The diagnosis of diabetes is not different because of the difference between adults and children, and the standards are the same.

### 3.2. Questionnaire Survey Method

Diabetic retinopathy is one of the most common fundus diseases. This is a general complication of diabetes and one of the main causes of blindness. Moreover, this disease is a staged cause. According to the recommendations of medical experts, diabetic patients need to be checked for diabetic retinopathy at least twice a year in order to detect signs of their illness in time. In the current clinical diagnosis, this disease mainly relies on the ophthalmologist's detailed examination of the color fundus images and then the evaluation of the patient's condition. Nowadays, the existing population is more than 1.3 billion. According to the statistical analysis of the World Health Organization's annual diabetes data, the current diabetes prevalence factors in the middle- and high-income groups are shown in Table 5:

As shown in Table 5, among diabetic patients, the ratio of males to females is similar, 12.4% for males, 8.4% for females, and fewer females than males. In obesity, 23.5% of men and 25.3% of women, women are higher than men, so in order to prevent diabetes, women should strengthen exercise.

Long-term diabetes leads to great changes in the microcirculation inside the retina, which is clinically manifested as various symptoms of pathological changes in the fundus. From a physiological point of view, it is believed that the blood sugar of diabetic patients tends to maintain a high level, which causes the red blood cells in the blood to carry and transmit the oxygen content which is greatly reduced compared with the normal level. Due to prolonged hypoxia, the capillary wall becomes thinner and weaker, resulting in microaneurysms.

In this paper, a comparative survey of men and women of different ages with diabetes is shown in Figure 8:

As shown in Figure 8, whether it is a high-age male or female, the probability of suffering from diabetes is about 3.8%, and the main factors affecting diabetes are as follows:

1. Genetic factors: according to statistics, both parents suffer from diabetes, and about 5% of children will have diabetes. If only one parent has diabetes, the children are less likely to suffer from diabetes. Diabetes is more affected by genetic inheritance and is a kind of genetic disease. People with relatives will be more likely to get the disease
2. Obesity factors: from 30 to 80 years old, muscle tissue gradually decreases, and body weight reduced from 45% to 34%, but fat increases from 17% to 33%. Obesity is the cause of the elderly, especially obese people, and one of the main causes of diabetes
3. Mental factors: when a person is in a state of high tension or excitement, there will be some stress reactions in the body. Human hormones, adrenal cortex hormones, and glucagon will increase to varying degrees, which leads to the secretion of hyperglycemic hormones. If things go on like this, it will easily lead to the development of diabetes and the aggravation of the symptoms
4. Lack of exercise: for a person who exercises regularly, the glycogen reserves and insulin secretion in the body are in regular fluctuations. The cells are also very sensitive to insulin, and the efficiency of rapid insulin response is high. When lack of exercise, the above situation is just the opposite. The occurrence of diabetes is from the decrease of sensitivity, decreased buffering capacity, or impaired glucose tolerance

Therefore, it can be seen from the analysis that long-term diabetes patients are more likely to develop lesions. It is very necessary to use medical big data to analyze the factors of patient prevalence. Medical big data can help to reasonably allocate scarce medical resources and improve the development of medical undertakings.

A cross-sectional survey was carried out, and patients were divided into two groups based on the presence or absence of clinical diabetic retinopathy. The physiological indicators of patients with diabetic retinopathy were tested and analyzed, and the inevitable relationship between the two was further investigated, as shown in Figure 9:

As shown in Figure 9, the prevalence of diabetic patients suffering from diabetic retinopathy is 47.5% in total. During diabetes, diabetic patients must strictly manage the urine albumin index, glycosylated hemoglobin index, and fasting blood glucose level, pay full attention to these risk factors, and manage these controllable influencing factors within the normal range.

Therefore, it is important to study the factor. Medical big data can reasonably allocate scarce medical resources to improve the quality of medical services. By rationally distributing medical resources, patients can get better medical and health services, which is conducive to promoting the development of the medical system. The emerging mobile medical system will profoundly change the traditional medical model. Medical big data has changed the way patients see a doctor. Patients can enjoy superior medical services without leaving their homes. The traditional medical service model with hospitals as the main body has undergone major changes.

## 4. Discussion

The medical data were used to analyze the causes of diabetic retinopathy. The relevant concepts of big medical data were explained and how to reduce the prevalence of diabetic retinopathy, through the questionnaire survey method case to discuss the importance of medical big data to contemporary society and finally take the medical big data into the survey of the prevalence of diabetic retinopathy to explore the correlation between the two.

This paper also makes reasonable use of the deeply supervised residual network algorithm based on medical big data. With the increasing application range of deep-supervised residual network algorithms and their importance gradually becoming more prominent, many scholars have begun to match the theory of deep-supervised residual network algorithms with real-life application scenarios and propose feasible algorithms. The deeply supervised residual network algorithm is a mathematical operation. According to this calculation, it is indispensable to investigate the main reasons that affect the prevalence of retinopathy in diabetic patients based on big medical data.

Through the questionnaire survey method, this article knows that according to medical big data, the conclusions drawn after investigating the main factors affecting the prevalence of retinopathy in diabetic patients are more accurate. Therefore, combining the characteristics of medical big data, find a new survey method, so that people can correctly and comprehensively understand the factors affecting the prevalence of retinopathy and how to prevent it.

## 5. Conclusions

This paper mainly introduces the theoretical knowledge of medical big data and the prevalence rate of patients' lesions and discusses how to use medical big data to investigate the influencing factors of patients' lesions. The deeply supervised residual network algorithm based on medical big data shows that in the process of applying deep supervision residual network algorithm to medical big data, good survey results can be obtained, and it lays a foundation for studying the factors affecting the prevalence of lesions. Moreover, the process is faster and more accurate, which has certain guiding significance for how to carry out the investigation of the factors affecting the prevalence of retinopathy in diabetic patients. Based on the wide range of related scientific fields involved in the medical big data research, the concept of medical big data has always been disputed, and the author's knowledge has not yet reached the perfect position. The author's academic theory and business ability are relatively weak, and there are still many deficiencies. At the same time, the author is constantly discovering and solving problems, striving to be the best.

## Figures and Tables

**Figure 1:** Schematic diagram of the deep supervision network structure.

**Figure 2:** Schematic diagram of the preactivated residual unit structure.

**Figure 3:** Processing a single image element in an artificial neural network.

**Figure 4:** Activation function graph.

**Figure 5:** Hyperplane and corresponding equation diagram.

**Figure 6:** Typical trajectory diagram.

**Figure 7:** Comparative analysis of sensitivity index and specificity of ensemble classifiers.

**Figure 8:** Comparison chart of men and women of different ages with diabetes.

**Figure 9:** Prevalence factors of retinopathy in diabetic patients.

**Table 1:** Network structure parameters of the deeply supervised residual network.

Network layer name	Filter size	Layer depth	Feature map size
Conv1	8∗8	1	220∗220
Conv2	9∗9	1	210∗210
Conv3	10∗10	0	111∗111
Conv4	11∗11	0	13∗13
Conv5	12∗12	3	24∗24
Conv6	13∗13	4	233∗333
Conv7	14∗14	3	143∗143
Conv8	15∗15	0	268∗268

**Table 2:** Classifier evaluation metrics table.

Measure	Formula
Accuracy (recognition rate)	TP + TN
Sensitivity (sensitivity)	TP/*P*
Specificity	TP + 1/*P*
Misjudgment rate	(TP/*P*) − 1
Yorden index	(TP/*P*) + TP − 1

**Table 3:** Accuracy of different ensemble learning methods at different scales under pruning.

	Scale 20	Scale 30	Scale 40	Scale 50
C4.5	86.654	98.644	95.543	97.864
Bagging+C4.5	84.865	98.432	98.644	98.315
Rotation Forest+C4.5	94.543	97.754	98.463	97.564
MultiBoostAB+C4.5	93.643	98.643	98.864	94.764
AdaboostM1+C4.5	94.532	93.754	98.342	96.574

**Table 4:** Accuracy of different ensemble learning methods at different scales without pruning.

	Scale 20	Scale 30	Scale 40	Scale 50
C4.5	87.754	92.542	94.242	97.321
Bagging+C4.5	94.643	98.613	97.632	99.521
Rotation Forest+C4.5	98.642	92.152	97.323	94.452
MultiBoostAB+C4.5	94.132	93.265	98.522	94.411
AdaboostM1+C4.5	94.656	98.732	94.238	98.743

**Table 5:** Diabetes prevalence factor table.

	Male	Female	Total
Diabetes	12.4%	8.4%	20.8%
Overweight	34.6%	23.6%	58.2%
Obesity	5.7%	6.7%	12.4%
Lack of exercise	23.5%	25.3%	48.8%

## Data Availability

No data were used to support this study.
